RETRACTED

# Bronchial blocker versus double-lumen endobronchial tube in minimally invasive cardiac surgery

**DOI:** 10.1186/s12890-019-0956-x

**Published:** 2019-11-09

**Authors:** Chuncheng Zhang, Jing Yue, Mingyue Li, Wei Jiang, Yu Pan, Zhimin Song, Cailian Shi, Weixuan Fan, Zhenxiang Pan

**Affiliations:** 1 Department of Anesthesiology, The Second Hospital of Jilin University, No.218 Ziqiang Street, Nanguan District, Changchun, 130041 Jilin province China; 2 Yanbian University, Yanbian, 130000 Jilin province China; 3 Department of Intensive Care Unit, The Second Hospital of Jilin University, Changchun, 130041 Jilin province China

**Keywords:** One-lung ventilation, Bronchial blocker, Double-lumen tube, Minimally invasive cardiac surgery, Cardiopulmonary bypass

## Abstract

**Background:**

To compare the therapeutic value of a bronchial blocker (BB) with a double-lumen tube (DLT) in minimally invasive cardiac surgery (MICS).

**Methods:**

Sixty patients who underwent MICS were randomized to use either a DLT (Group D, *n* = 30) or a BB (Group B, *n* = 29; one failed was omitted). The following data were collected: time of intubation and tube localization; incidence of tube displacement; postoperative sore throat and hoarseness; time of cardiopulmonary bypass; maintenance time for SpO_2_ < 90% (PaCO_2_ < 60 mmHg); mean arterial pressure and heart rate; SpO_2_, PaO_2_, PaCO_2_, EtCO_2_, mean airway pressure, and airway peak pressure; surgeons’ satisfaction with anesthesia; and short-term complications.

**Results:**

The times of intubation and tube localization were significantly longer in Group B than in Group D (*P* < 0.05). Patients in Group B exhibited significantly lower incidence of tube displacement, postoperative sore throat, and hoarseness when compared with patients in Group D (*P* < 0.05). Mean arterial pressure and heart rate were significantly lower in Group B than in Group D after tracheal intubation (*P* < 0.05). The mean airway pressure and airway peak pressure were significantly lower in Group B than in Group D after one-lung ventilation (*P* < 0.05). SpO_2_ and PaO_2_ in Group B were significantly higher than in group D after cardiopulmonary bypass (*P* < 0.05). No short-term postoperative complications were observed in patients of Groups B and D during 3 month follow-up.

**Conclusion:**

BB can be a potential alternative to the conventional DLT for lung isolation in MICS. Trial registration: ChiCTR1900024250, July 2, 2019.

## Background

Minimally invasive cardiac surgery (MICS) is a kind of heart surgery performed through a mini-thoracotomy [1]. MICS is widely applied in clinical practice, due to its advantages of minimal trauma, less postoperative pain, short hospital stay, and fast recovery [2].

RETRACTED

Lung isolation is needed to meet the exposure of the surgical field and evaluation of pulmonary function during MICS [3]. The use of a double-lumen tube (DLT) is one of the most commonly utilized strategies in lung isolation [4]. The use of a DLT results in a low risk of movement after positioning, and allows for continuous positive airway ventilation to the deflated lung. A bronchial blocker (BB), a device which can be inserted down a tracheal tube after tracheal intubation, can also meet the needs of lung isolation [5]. Until now, the choice between DLT and BB is still controversial, and conflicting results have been revealed [6–8]. It has been reported that neither left-sided DLT or Arndt® wire-guided blocker (Cook Medical, Bloomington, IN, USA) during intubation offered any significant advantages in morbidly obese patients [6]. A BB with spontaneous collapse takes longer to deflate and does not provide equivalent surgical exposure compared to a DLT in patients undergoing elective pneumothorax surgery [7]. A Y-shaped BB, EZ-Blocker (Teleflex Life Sciences Ltd., Athlone, Ireland) is an efficient and effective device for lung isolation, and causes less injury and sore throat compared with a DLT [8]. However, to our knowledge, there is still no study on the application of BB in MICS with cardiopulmonary bypass (CPB) and its outcomes when compared with using a DLT.

In this study, patients undergoing MICS were enrolled, and the clinical values relating to the use of BB and DLT were evaluated and compared. Our findings reveal an effective and safe strategy in maintaining lung isolation during MICS with CPB.

## Methods

### Patients

A total of 60 patients (33 male, 27 female; 30–65 years old) in need of mitral/tricuspid valve replacement or annuloplasty (MICS) were recruited from the Department of Cardiothoracic Surgery in the Second Hospital of Jilin University from December 2012 to February 2016.

The inclusion criteria were as follows: i) patients had mitral/tricuspid insufficiency; ii) patients had symptomatic and moderate-to-severe mitral stenosis; iii) patients had chronic and severe mitral regurgitation (cardiac function New York Heart Association or NYHA grade II-III) without severe left ventricular dysfunction (ejection fraction < 0.30) and/or systolic late diameters > 55 mm; iv) patients had asymptomatic chronic severe mitral regurgitation, mild-to-moderate left ventricular dysfunction (ejection fraction of 0.30–0.60) and/or systolic late diameter ≥ 40 mm; v) unable to perform percutaneous balloon mitral valvuloplasty; vi) American Society of Anesthesia (ASA) grade IIs-III. The exclusion criteria were additional contraindications for lung isolation and MICS, such as acute airway inflammation, laryngeal edema, tracheal compression, and coagulation dysfunction.

RETRACTED

All enrolled patients were randomly divided into the DLT group (Group D) and the BB group (Group B). All patients and their families were fully informed of the purposes and procedures of this study, as well as the potential intra- and postoperative complications. Informed written consent was obtained from all participants and their relatives. This study was approved by the Ethics Committee of the Second Hospital, Jilin University.

### Surgical procedure

#### Lung isolation

Lung isolation was performed before opening of the pleura. The conditions of lung isolation were as follows: the pressure inside the sleeve capsule of the left tube was low, between 15 and 20 cm; the volume inside the sleeve capsule was 2-3 ml; and auscultation of isolated lung respiratory tone disappeared. Because arterial blood pressure and heart rate might increase temporarily after anesthesia induction, the tracheal intubation was implemented at 5 min after anesthesia induction with 0.1 mg/kg imidazole, 0.05 mg/kg midazolam, 1.5–2 μg/kg sufentanil and 0.1 mg/kg vecuronium. DLT was inserted into patients of Group D, and the tube position was confirmed by flexible bronchoscopy (FOB) (Olympus BF-240 bronchoscope; Olympus America, Pennsylvania, USA) in left semi-lateral position at 45 degree. Meanwhile, single lumen tube combined with a BB (Tappa Medical Technology Co., Ltd., Hangzhou, China) was inserted into patients of Group B, and positioned under FOB guidance in the operative position. Notably, tube displacement was detected by fiberoptic bronchoscopy after left semi-lateral position at 45 degree, and the best position of the tube was adjusted by means of fibronchoscopy.

A 7.5–8 ^#^ tracheal tube (Mallinckrodt™ Lo-Contour Oral/Nasal T real Tube Cuffed, Mallinckrodt Hi-Lo (TM), Covidien, Dublin, Ireland) or a 37 ^#^/39 ^#^ left DLT (Mallinckrodt™ Endobronchial Tube) was selected in male patients, while a 7–7.5 ^#^ tracheal tube or 35 ^#^/37 ^#^/39 ^#^ left DLT was used in female patients. In group D, 35 ^#^, 37 ^#^, and 39 ^#^ DLTs were used in 10, 11, and 9 patients, respectively. In Group B, 7 ^#^, 7.5 ^#^, and 8 ^#^ single lumen tubes were used in 9, 16, and 4 patients, respectively.

Transesophageal echocardiography was performed after completing intubation, and mechanical ventilation was set in the volume-controlled ventilation model at 8–10 ml/kg of ideal body weight with 95% oxygen concentration. Once the ascending aorta was blocked, oxygen supply was stopped, and the tracheal tube cuff was deflated. Oxygen supply was regained by one-lung ventilation after removing the blockage. When the SpO_2_ became < 90% (PaCO_2_ < 60 mmHg), the cuff of the BB in Group B was partially relaxed, and the right lung was expanded to meet the gas exchange requirement. When removing the BB after the surgery, the tracheal tube was pulled out as appropriate. In Group D, double lung ventilation was performed until SpO_2_ was > 90% (PaCO_2_ > 60 mmHg). The surgery was performed under single lung ventilation. After the surgery, the DLT in Group D was replaced with a single-lumen tracheal tube using a tube exchanger or a direct laryngoscop.

RETRACTED

#### MICS

CPB was maintained after lung isolation. For mitral valve surgery, the aorta was clamped, cardiac arrest was induced by perfusion of cardioplegia, and the oxygen supply was stopped. When valve replacement was completed, the left atrium was closed, the clamped aorta was released, and the oxygen supply returned. Aortic blockage was not need for tricuspid valve surgery. Before closing of the chest, the patient was weaned off CPB, and double lung ventilation was performed.

#### Outcome measurements

The primary outcome was arterial oxygen partial pressure (PaO_2_). Other outcomes were also collected, including: 1) the times of intubation and tube localization; 2) the incidences of tube displacement (> 1.5 cm was defined as a significant displacement), 3) postoperative sore throat, and hoarseness; and 4) the mean arterial pressure (MAP) and heart rate (HR) before and after intubation; 5) the time of cardiopulmonary bypass (CPB); 6) maintenance time (T) for SpO_2_ < 90% (PaCO_2_ < 60 mmHg); 7) peripheral oxygen saturation (SpO_2_), PaCO_2_, EtCO_2_, and mean airway pressure and airway peak pressure before (T1) and 30 min after (T2) one-lung ventilation, 30 min after CPB (T3), and 30 min before (T4) the end of the operation; and 8) surgeons’ satisfaction with anesthesia that were evaluated by the same surgical surgeon.

Patients were followed-up for 3 months after the surgery, and the occurrence of short-term complications were recorded, such as peritoneal leakage, artificial valve thrombosis, thromboembolism, acute respiratory failure, hepatic insufficiency, low cardiac output syndrome, and multiple organ failure.

#### Statistical analysis

SPSS 18.0 software (SPSS Inc., Chicago, IL, USA) was used for statistical analysis. The sample size was conducted using Power analysis and sample size (PASS) software package program (Utah, USA, version 11.0 for windows). Continuous variables were expressed as mean ± standard deviation (SD), and categorical variables as percentages. Differences between different groups were compared using t-test for continuous variables, and chi-square (*χ*^*2*^)-test for categorical variables.

RETRACTED

## Results

The Non-Inferiority Tests for Two Means [Differences] in the SPSS was used to calculate the sample size, with the Power = 0.9, α = 0.025, clinically meaningful expected difference = 15 mmHg. Two groups of sample size ratio of 1:1 and the sample size was 20 individuals per group. The result indicated that there were sufficient sample sizes to obtain significant differences in PaO2 between the two groups. There was one case in Group B group, who underwent three times of BB intubation, all of which were entered into the right main bronchus. Considering the effect on surgical conditions, this case was given up in this study and received DLT for treatment. Except for one failed BB intubation, MICS was successfully performed in 30 patients in Group D and 29 patients in Group B. The results showed that BB had a 3.3% (1/30) failure rate compared to 0% failure rate of DLT in terms of placement. No significant differences were revealed with regard to the age, gender, height, and weight between Groups D and B (*P* > 0.05) (Table 1).

**Table 1:** Clinical characteristics of patients receiving double-lumen tube (DLT) (Group D) and bronchial blocker (BB) (Group B)

Data	Group D (*n* = 30)	Group B (*n* = 29)	*P*
Age (year)	45 ± 7	46 ± 8	0.897
Gender (male/female)	18/12	16/13	0.708
Weight (kg)	62.3 ± 9.3	65.9 ± 8.4	0.812
Height (cm)	168.5 ± 5.9	169.4 ± 6.3	0.893
Intubation time (min)	8.5 ± 3.5	9.6 ± 4.9	0.035
Time of tube location (min)	13.6 ± 4.2	15.5 ± 4.3	0.023
Tube displacement (%)	18.0	4.2	0.037
Lung collapse (no/partial/complete)	23/7/0	26/3/0	0.184
Anesthesia satisfaction (%)	90 ± 3	97 ± 1	0.053
T (SpO_2_ < 90%) (min)	10.3 ± 2.1	11.1 ± 1.9	0.892
CPB time (min)	97.2 ± 34.5	95.7 ± 32.3	0.769
Postoperative sore throat (%)	53.3	17.2	0.004
Postoperative hoarseness (%)	13.3	3.4	0.013

*CPB* cardiopulmonary bypass; T: maintenance time for SpO_2_ < 90% (PaCO2 < 60 mmHg) after CPB

The times of intubation and tube localization were significantly longer in Group B than in Group D (intubation: 8.5 ± 3.5 min vs. 9.6 ± 4.9 min, *P* = 0.035; tube localization: 13.6 ± 4.2 min vs. 15.5 ± 4.3 min, *P* = 0.023). Patients in Group B exhibited significantly lower incidence of catheter displacement (4.2% vs. 18.0%, *P* = 0.037), postoperative sore throat (18.2% vs. 53.3%, *P* = 0.004), and hoarseness (0.34% vs. 13.3%, *P* = 0.013) when compared to patients in Group D. There were no statistical differences found in CPB time, T, lung collapse, and anesthesia satisfaction between Groups D and B (*P* > 0.05) (Table 1).

The hemodynamics of patients in Groups B and D were noted before and after tracheal intubation. As shown in Table 2, no significant differences in MAP and HR were observed between these groups before tracheal intubation. However, MAP (*P* = 0.035) and HR (*P* < 0.001) were significantly lower in Group B than in Group D after tracheal intubation.

RETRACTED

**Table 2:** The hemodynamics of patients receiving double-lumen tube (DLT) (Group D) and bronchial blocker (BB) (Group B) before and after tracheal intubation

Data	Group D (*n* = 30)		Group B (*n* = 29)	
	Before	After	Before	After
MAP (mmHg)	64 ± 12	80 ± 16	63 ± 14	75 ± 10^*^
HR (beats/min)	87 ± 9	100 ± 9	85 ± 10	90 ± 5^*^

*MAP* Mean arterial pressure, *HR* Heart rate. *P < 0.05 vs. Group D

As shown in the Table 3, the oxygenation index and airway pressure of patients in Groups B and D were further evaluated at different time points. After one-lung ventilation, patients in Group B exhibited significantly lower mean airway pressure and airway peak pressure than those in Group D (T2, T3, and T4) (*P* < 0.05). After CPB, SpO_2_ and PaO_2_ in Group B were significantly higher than those in Group D (T3 and T4) (*P* < 0.05). No statistical differences were revealed in PaCO_2_ and EtCO_2_ between these two groups.

**Table 3:** Oxygenation index and airway pressure of patients receiving double-lumen tube (DLT) (Group D) and bronchial blocker (BB) (Group B) at different time points

	Group D (*n* = 30)				Group B (*n* = 29)			
	T_1_	T_2_	T_3_	T_4_	T_1_	T_2_	T_3_	T_4_
SpO_2_ (%)	99 ± 1	99 ± 1	94 ± 4	98 ± 1	98 ± 2	99 ± 1	98 ± 1^*^	99 ± 1^*^
PaO_2_ (mmHg)	134.4 ± 9.4	145.3 ± 10.2	99.2 ± 9.8	120.3 ± 9.4	135.2 ± 8.9	143.3 ± 11.2	119.3 ± 8.9^*^	137 ± 8.4^*^
PaCO_2_ (mmHg)	42.2 ± 4.2	42.6 ± 6.5	45.1 ± 4.2	41.2 ± 2.4	43.4 ± 4.8	43.4 ± 6.5	44.4 ± 5.2	40.5 ± 3.5
EtCO_2_ (mmHg)	36.8 ± 4.5	37.2 ± 4.1	34.6 ± 5.1	31.7 ± 4.7	35.5 ± 6.1	36.3 ± 5.8	36.5 ± 4.8	32.1 ± 5.3
Ppeak (cmH_2_O)	20.0 ± 3.2	27.0 ± 3.3	29.2 ± 3.4	27.6 ± 3.0	19.2 ± 2.2	24.5 ± 3.5^*^	26.5 ± 2.3^*^	25.3 ± 2.7^*^
Pmean (cmH_2_O)	7.0 ± 2.1	9.0 ± 1.8	9.3 ± 2.0	8.9 ± 2.1	6.0 ± 1.5	8.3 ± 1.7^*^	8.5 ± 1. 6^*^	8.1 ± 1.8^*^

Ppeak: airway peak pressure; Pmean: mean airway pressure; T_1_: before one lung ventilation; T_2_:30min after one lung ventilation; T_3_:30min after cardiopulmonary bypass; T_4_: 30 min before the operation end. ^*^P < 0.05 vs. Group D

During the follow-up of 3 months, no short-term postoperative complications were observed in patients of both Groups B and D. No death occurred in the 59 participants.

## Discussion

Pulmonary insufficiency is one of the earliest recognized complications of cardiac surgery [9]. The use of BB and DLT has been widely applied in thoracic surgery [10], while the application of BB in MICS with CPB has not been reported. To our knowledge, this is the first study to assess the feasibility of BB use in MICS with CPB, as compared to the use of DLT.

RETRACTED

In this study, we found that the intubation time and tube localization time of Group B were significantly longer than those of Group D. Our finding is consistent with previous studies. It has been reported that DLT is quicker to place and less likely to be incorrectly positioned than BB [11]. A single-lumen tube combined with BB requires more laryngoscopy attempts and additional time to replace than a DLT [12]. However, a DLT has to be replaced by a single-lumen tube to maintain postoperative mechanical ventilation after surgery. Patients receiving a BB only need to pull out the bronchial occluder. We suspect that the extra minute for the entire intubation process using a BB is negligible. The use of a BB cannot be abandoned by relying solely on this data in clinic practice.

Since the use of a BB exhibits less damage on the trachea, some researchers prefer to use a BB in lung isolation. It has been reported that a BB is associated with a low incidence of airway injury and a low severity of injury [11]. A Y-shaped BB is easier for one-lung ventilation, and causes less injury and sore throat than a DLT [8]. Consistent with these findings, our study found that the incidence of sore throat and hoarseness were both significantly lower in patients for whom a BB was used compared to those for whom a DLT was used. This result may be explained by the fact that the outside diameter of a DLT is larger than that of single-lumen tube with the same inner diameter [13]. When the outside diameter is consistent, the airway pressure of a BB is lower than that of a DLT after single-lung ventilation. Small airway resistance favors the redistribution of pulmonary blood flow to the ventilated lung, thus relieving intrapulmonary shunting and improving oxygenation during single-lung ventilation [14].

MAP and HR are important indicators of intubation safety. In this study, we found that MAP and HR were significantly lower in Group B than in Group D after tracheal intubation. The relatively small changes of MAP and HR indicate that BB can be safely applied to patients undergoing cardiac surgery. Ender et al. [15] reported that single-lung ventilation can reduce PaO_2_/FIO_2_ by 62 to 70% in MICS. In the present study, significantly higher SpO_2_ and PaO_2_ were revealed in Group B than in Group D after CPB. This result may be explained by the fact that the application of BB can relieve the systemic inflammatory response on pulmonary function after CPB.

In summary, although more time is spent on intubation and tube localization, a BB appears to be more suitable for lung isolation in MICS with CPB compared to a DLT. This study, however, is still limited by an insufficient population, and the enrolled patients are all ASA II-III. Meanwhile, BB had a 3.3% (1/30) failure rate compared to 0% failure rate of DLT in terms of placement, which might influence clinical application of BB to some extent. Lastly, we did not record the incidence of prolonged intubation post operation, which would affect the rate of postoperative sore throat and hoarseness. Further researches on the application of BBs based on a large population and complete design are still needed.

RETRACTED

## Conclusion

A BB can effectively and safely maintain lung isolation, and thus can be a potential alternative to the conventional DLT in MICS.

## Data Availability

Not applicable. This study was only the primary research, and further study is in progress.

## Abbreviations

ASA: American Society of Anesthesia
BB: Bronchial blocker
CPB: Cardiopulmonary bypass
DLT: Double-lumen tube
HR: Heart rate
MAP: Mean arterial pressure
MICS: Minimally invasive cardiac surgery
